# Prediction of Outlet Pressure for the Sulfur Dioxide Blower Based on Conv1D-BiGRU Model and Genetic Algorithm

**DOI:** 10.1155/2022/6297746

**Published:** 2022-09-27

**Authors:** Xiaoli Li, Chengzhong Xu, Kang Wang, Zhiqiang Liu, Guihai Li

**Affiliations:** ^1^Faculty of Information Technology, Beijing University of Technology, Beijing 100124, China; ^2^Beijing Key Laboratory of Computational Intelligence and Intelligent System, Beijing University of Technology, Beijing 100124, China; ^3^Engineering Research Center of Digital Community, Beijing University of Technology, Beijing 100124, China; ^4^Guixi Smelter, Jiangxi Copper Corporation Limited, Guixi, Jiangxi 335400, China; ^5^Beijing RTlink Technology Co. Ltd., Beijing 100024, China

## Abstract

The sulfur dioxide blower is a centrifugal blower that transports various gases in the process of acid production with flue gas. Accurate prediction of the outlet pressure of the sulfur dioxide blower is quite significant for the process of acid production with flue gas. Due to the internal structure of the sulfur dioxide blower being complex, its mechanism model is difficult to establish. A novel method combining one-dimensional convolution (Conv1D) and bidirectional gated recurrent unit (BiGRU) is proposed for short-term prediction of the outlet pressure of sulfur dioxide blower. Considering the external factors such as inlet pressure and inlet flow rate of the blower, the proposed method first uses Conv1D to extract periodic and local correlation features of these external factors and the blower's outlet pressure data. Then, BiGRU is used to overcome the complexity and nonlinearity in prediction. More importantly, genetic algorithm (GA) is used to optimize the important hyperparameters of the model. Experimental results show that the combined model of Conv1D and BiGRU optimized by GA can predict the outlet pressure of sulfur dioxide blower accurately in the short term, in which the root mean square error (RMSE) is 0.504, the mean absolute error (MAE) is 0.406, and R-square (*R*^2^) is 0.993. Also, the proposed method is superior to LSTM, GRU, BiLSTM, BiGRU, and Conv1D-BiLSTM.

## 1. Introduction

With the rapid development of the industrial process, the demand for energy and materials has been increasing, especially for nonferrous metals. Therefore, the smelting of nonferrous metals is also gradually increasing. However, nonferrous metals often exist in nature in the form of sulfide. As a result, a large amount of flue gas containing sulfur dioxide is produced in the smelting process. If the flue gas is directly discharged into the environment, there will be serious problems such as air pollution and soil acidification. To protect the environment, it is necessary to recover sulfur dioxide from flue gas in metal smelters. Acid production with flue gas is the most widely used and technically most mature desulfurization process at present. The system of acid production with flue gas is inseparable from the blower that transports the flue gas. The outlet pressure of the blower affects the flue gas desulfurization process and, more importantly, the conversion rate of sulfur dioxide into sulfuric acid [1]. How to predict the outlet pressure of the blower in the process of acid production with flue gas and improve its prediction accuracy is the main research work.

For the problem of pressure prediction of time series data, many scholars in the world have proposed a lot of methods. The analytical methods at the present of pressure prediction are divided into two main categories: classical time series models based on mathematics and statistical theory and prediction models based on machine learning [2]. The traditional time series models are AR, ARMA, ARIMA, etc. However, the traditional time series models have many limitations on the data. Most of them are only applicable to the smooth time series, and a series of operations such as normalization and differencing are needed for the nonsmooth data. Meanwhile, it is difficult to predict the sudden changes in the time series [3]. Machine learning and deep learning forecasting algorithms are widely used in time series forecasting problems in recent years due to easier data processing and good nonlinear and multivariate forecasting capabilities [3, 4]. Yu et al. [5] proposed four machine learning algorithms to predict void pressure using a multilayer perceptron neural network, support vector machine, random forest, and gradient augmentation machine. Random forest outperformed other machine learning algorithms in terms of goodness of fit, generalization, and prediction accuracy, but the random forest was prone to overfitting problems. Liu et al. [6] used a multilayer feedforward artificial neural network (ANN) for failure pressure prediction. By comparing the experimental blast test results and the results of previous failure pressure estimation models, the ANN model results were demonstrated to be highly accurate and efficient. Zhao et al. [7] proposed a blood pressure prediction model based on a long short-term memory (LSTM) network. Also, the model made full use of the efficient processing properties of the LSTM for time series information to accurately predict systolic and diastolic blood pressure. Song et al. [8] used an LSTM model instead of a conventional pressure sensor to sense the differential pressure in the gas turbine intake filter and verified its high virtual sensing accuracy and model portability. Gao et al. [9] combined a new cost function (relative mean square error) with a gated recurrent unit (GRU) to propose an earth pressure prediction model and obtained better prediction results. Wang et al. [10] used the CNN-GRU model for multivariate prediction of water pipe network pressure and achieved better performance but did not consider the contextual relationship of data.

Although domestic and foreign researchers have proposed many worthwhile methods for the pressure prediction problem, some aspects have not been taken into consideration. First, most pressure prediction methods use only historical data of pressure without considering the influence of external factors and do not explore the correlation characteristics and period characteristics among them. Second, some methods ignore the contextual relationship of these data, and the prediction accuracy is reduced [11]. Third, many prediction models have complex parameter settings and in many cases are not set to the optimal parameter combination. Fourth, the convergence of the model is slow, resulting in a slow experimental process. Considering the above discussion, a novel model combining Conv1D-BiGRU and GA for sulfur dioxide blower's outlet pressure prediction is proposed. Conv1D is used to extract the horizontal relationship features of multidimensional variables before BiGRU [12]. BiGRU is used to learn the temporal relationship of the features extracted by Conv1D [13]. GA is used to find the optimal parameters of the Conv1D-BiGRU model [14]. The multivariable spatial features are convolved in the model and then added to the GRU network for bidirectional extraction of temporal features. Multivariable time series data can be handled well by it. Meanwhile, GA is used to optimize the parameters of Conv1D-BiGRU to further improve the prediction performance. It is verified that the proposed method can be used well for outlet pressure prediction of sulfur dioxide blower. The system architecture of this study is shown in Figure 1.

The whole research process combines artificial neural network and optimization algorithm. It involves neural network modeling, neural calculation, and neural network optimization. The artificial neural network uses the Conv1D network and BiGRU network, which involves the long short-term memory of time series. Then, GA is used to optimize the hyperparameters of artificial neural network. The optimized artificial neural network is used to predict the time series. This research belongs to the field of neural network modeling, neural computation, and network optimization. The rest of the arrangement is as follows.  Section 2 presents related work, including an introduction to the process of acid production with flue gas and the principles of the relevant models.  Section 3 presents model construction and hyperparameter optimization based on GA.  Section 4 presents experiments and analysis, including a comparison of the proposed model with other models.  Section 5 presents conclusions and an outlook.

## 2. Related Work

This section introduces the process flow of the system of acid production with flue gas and clarifies the significance of the sulfur dioxide blower. The principles of Conv1D, LSTM, GRU, and BiGRU are introduced. In addition, the current research status of the Conv1D-BiGRU model and optimization algorithm is also introduced.

### 2.1. Analysis of Acid Production Process with Flue Gas

The acid production system with flue gas is studied based on a smelter in Jiangxi Province. The process of acid production with flue gas at the smelter is currently using a single-stage centrifugal blower with an adjustable guide vane, as shown in Figure 2. The flue gas from copper smelting is sent to the blower after the purification section and the dry suction section, so the blower is also known as a sulfur dioxide blower. The flue gas after treatment is fed into the conversion section through the sulfur dioxide blower. Sulfur dioxide goes through the conversion process and reacts to produce sulfuric acid in different concentrations. The whole process of acid production with flue gas is shown in Figure 3. The prediction and control of the outlet pressure of the sulfur dioxide blower are crucial to the acid production process. Too heavy outlet pressure will lead to flue gas leakage; however, too less outlet pressure will form negative pressure and damage the equipment. The outlet pressure also affects the conversion rate of SO_2_ to SO_3_. However, owing to the complex internal structure of the blower and the uncertainty of the external disturbance, it is difficult to predict the outlet pressure of the blower.

### 2.2. One-Dimensional Convolution (Conv1D)

Convolutional neural networks (CNNs) have achieved a series of breakthrough research results in the fields of image classification, target detection, and semantic segmentation of images [15]. The powerful feature learning and classification capabilities have attracted widespread attention. CNN is a typical feedforward neural network, which essentially extracts the features of the input data by building multiple filters. These filters convolve and pool the input data layer by layer to extract the topological features embedded in the input data. A typical CNN usually consists of an input layer, a convolutional layer, a pooling layer, a fully connected layer, and an output layer, as shown in Figure 4. In the convolutional layer, the convolutional kernel convolves the feature vector of the previous layer, and the output feature vector is constructed by using a nonlinear activation function. The input of a 1D CNN is 1D data, so its convolution kernel is also 1D structured accordingly. Also, the output of each convolutional and pooling layer is a 1D feature vector accordingly. The low-dimensional information of time series can be well extracted by using Conv1D, whose mathematical model can be described as follows:

(1) $$\begin{array}{c} y\left(k\right)=h\left(k\right)*u\left(k\right)=\overset{N}{\underset{i=0}{\sum }}h\left(k-i\right)u\left(i\right)\text{,} \end{array}$$

where *y*(*k*) denotes the function used for the convolution calculation, *h*(*k*) and *u*(*k*) denote the input and convolution kernel, respectively, *k* is the kernel size, and *i* denotes the index of the data in the sequence.

### 2.3. Long Short-Term Memory (LSTM)

Among many deep learning models, recurrent neural network (RNN) introduces the concept of temporal order into the network structure design, which makes it more adaptable in temporal data analysis. The basic idea of RNN is gradient backpropagation over time. However, in the process of backpropagation over time, the gradient of subsequent nodes will deviate from the initial value due to the too deep network or inappropriate activation function. Hence, it is prone to gradient disappearance and gradient explosion problems [16]. To solve this problem, LSTM was born as a classical variant of RNN, and the structure of a single neuron of LSTM is shown in Figure 5.

The computational principle of LSTM can be explained by the following equations.

(2) $$\begin{array}{c} f_{t}=\sigma \left(w_{f}x_{t}+u_{f}h_{t-1}+b_{f}\right)\text{,} \end{array}$$

(3) $$\begin{array}{c} i_{t}=\sigma \left(w_{i}x_{t}+u_{i}h_{t-1}+b_{i}\right)\text{,} \end{array}$$

(4) $$\begin{array}{c} o_{t}=\sigma \left(w_{o}x_{t}+u_{o}h_{t-1}+b_{o}\right)\text{,} \end{array}$$

(5) $$\begin{array}{c} \tilde{c_{t}}=\tanh\;\left(w_{c}x_{t}+u_{c}h_{t-1}+b_{c}\right)\text{,} \end{array}$$

(6) $$\begin{array}{c} c_{t}=f_{t}\cdot c_{t-1}+i_{t}\cdot \tilde{c_{t}}\text{,} \end{array}$$

(7) $$\begin{array}{c} h_{t}=o_{t}\cdot \;\tanh\left(c_{t}\right)\text{.} \end{array}$$

Figure 5 and equations (2)–(7) show that the LSTM consists of four parts: input gate, memory unit, output gate, and forgetting gate. *x*_*t*_ denotes the input vector at time *t*, *h*_*t − *1_ denotes the output vector at the previous time, *w*_*i*_, *w*_*o*_, *w*_*c*_ denote the weight coefficient matrix of each corresponding part, *b*_*f*_, *b*_*i*_, *b*_*o*_, *b*_*o*_ denote the offset vector of each corresponding part, *σ* denotes the activation function sigmoid, *f*_*t*_ is the value of the forgetting gate, which indicates how much information needs to be forgotten, *i*_*t*_ is the value of the input gate, which indicates how much candidate memory information needs to be saved, $\tilde{c_{t}}$ denotes the value of the candidate memory cell, *c*_*t*_ denotes the value of the memory cell jointly determined by *i*_*t*_ and $\tilde{c_{t}}$, and *o*_*t*_ is the value of the output gate, which controls how much information *c*_*t*_ outputs to the output vector *h*_*t*_.

### 2.4. Gated Recurrent Unit (GRU)

With the widespread use of LSTM in natural language processing and temporal sequences, the shortcomings of LSTM networks with long training times and numerous internal parameters need to be addressed urgently. A variant of LSTM, GRU, was subsequently proposed. The GRU consists of only update gates and reset gates. Meanwhile, the GRU model not only maintains the advantages of LSTM but also features a simpler structure, fewer parameters, and better convergence [17]. The specific structure of a single neuron is shown in Figure 6.

The principle of GRU can be explained by the following equations.

(8) $$\begin{array}{c} r_{t}=\sigma \left(w_{r}x_{t}+u_{r}h_{t-1}+b_{r}\right)\text{,} \end{array}$$

(9) $$\begin{array}{c} z_{t}=\sigma \left(w_{z}x_{t}+u_{z}h_{t-1}+b_{z}\right)\text{,} \end{array}$$

(10) $$\begin{array}{c} {\tilde{h}}_{t}=\tanh\;\left(w_{h}x_{t}+u_{h}\left(r\cdot h_{t-1}\right)+b_{h}\right)\text{,} \end{array}$$

(11) $$\begin{array}{c} h_{t}=z_{t}\cdot h_{t-1}+\left(1-z_{t}\right)\cdot \tilde{h_{t}}\text{,} \end{array}$$

where *σ* denotes the activation function sigmoid, *r*_*t*_ denotes the reset gate at time *t*, *z*_*t*_ denotes the update gate at time *t*, $\tilde{h_{t}}$ denotes the candidate activation state at time *t*, *h*_*t*_ denotes the activation state at time *t*, and *h*_*t − *1_ denotes the hidden state at time *t* − 1. The GRU has a more streamlined structure, which improves training efficiency to a large extent.

### 2.5. Bidirectional Gated Recurrent Unit (BiGRU)

Both the traditional LSTM and GRU pass information from forward to backward, which has limitations in many tasks and does not fully exploit the data information. To solve this problem, two forward and backward GRU networks, called BiGRU, are designed. The idea of BiGRU is to connect the same input sequence into two GRUs, forward and backward, respectively. Then, the implicit layers of the two networks are connected to the output layer for prediction [18]. Its structure is shown in Figure 7.

The BiGRU model is a neural network consisting of two GRU hidden layers together, which receive the same input at each moment. But the two hidden layers are in opposite directions, which can improve the accuracy and depth of feature vector extraction. The principle of the BiGRU model can be explained by the following equations.

(12) $$\begin{array}{c} \overset{⟶}{h_{t}}=GRU\left(x_{t},\overset{⟶}{h}{}_{t-1}\right)\text{,} \end{array}$$

(13) $$\begin{array}{c} \overset{\leftarrow }{h}{}_{t}=GRU\left(x_{t},\overset{\leftarrow }{h}{}_{t-1}\right), \end{array}$$

(14) $$\begin{array}{c} h_{t}=w_{t}\overset{⟶}{h_{t}}+v_{t}\overset{\leftarrow }{h}{}_{t}+b_{t}, \end{array}$$

where the *GRU*(.) function represents a nonlinear transformation of the input time data, *x*_*t*_ is the input, $\overset{⟶}{h_{t}}$ is the forward hidden state output, $\overset{\leftarrow }{h}{}_{t}$ is the reverse hidden state output,*w*_*t*_ denotes the weight corresponding to the forward hidden state at time *t*, *v*_*t*_ denotes the weight corresponding to the reverse hidden state, and *b*_*t*_ denotes the bias corresponding to the BiGRU double hidden state at time *t*.

In this study, the Conv-BiGRU model and an optimization algorithm are combined. The recent related studies were analyzed. Wang et al. [19] proposed a multitask learning (MTL) classification method based on the CNN-BiGRU model for improving the accuracy and efficiency of legal decision prediction. However, the model is mainly used for text classification and our task is time series prediction. Arshad et al. [20] proposed the CNN-BiGRU model to improve the accuracy of gait event detection in the elderly. However, this model uses data from a single sensor and this paper's target data are from multiple sensors. Joolee et al. [21] used the Conv1D-BiGRU model to understand the tactile sensation of real objects from haptic data, but the model is useful for classification and not for regression analysis. Lakshmanna et al. [22, 23] used frequent DNA sequence mining using optimization (FDSMO) which combines frequent biological sequence based on bitmap (FBSB) and hybrid of firefly and group search optimization (HFGSO) for DNA sequence mining. Subsequently, a novel DNA sequence mining method based on multiple constraints with HFGSO is proposed. Higher quality results were obtained. But these methods are more applicable to DNA sequences than to time series. Kara [24] used a hybrid method that combines LSTM neural network and GA for multistep influenza outbreak forecasting problems. Although a good prediction effect was achieved, the spatial characteristics among the multivariable were not considered. The combination of Conv1D-BiGRU model and GA proposed in this paper can be well applied to the prediction of multivariate time series.

## 3. Methodology

To improve the prediction accuracy of sulfur dioxide blower outlet pressure, Conv1D and BiGRU are combined to obtain a more in-depth and excellent model. The proposed model can accurately predict the future information of the outlet pressure of the sulfur dioxide blower based on various historical data. In Section 3.1, the model structure of Conv1D-BiGRU is introduced and the design principles of the model are elaborated. In Section 3.2, the process of setting the hyperparameters of the model using GA is described.

### 3.1. The Model Based on Conv1D and BiGRU

The proposed model is a combination of Conv1D and BiGRU. The model consists of an input layer, a convolutional layer, a BiGRU layer, a dropout layer, a fully connected layer, and an output layer. The input layer can receive multivariate sequence data. The Conv1D layer can obtain the features of the sequence by convolutional computation of the sequence data and convolutional kernel. It can also shorten the length of the sequence and enhance the dependency between the data. The BiGRU layer can effectively capture the information association between long sequence contexts by two one-way GRUs with the same input and the opposite direction of information transfer and mitigate the gradient disappearance or explosion. The dropout layer can remove the units of the BiGRU layer from the network with a certain probability to reduce overfitting. The fully connected layer is the sensing layer, which is responsible for mapping the features to the sample space. The output layer is responsible for outputting the sequence data at the same latitude as the sample space. The specific structure is shown in Figure 8.

Next, the computational logic and construction principle of the model are elaborated. Imagine a set of time series data with time step *n* and feature number *f*, as shown in the following equation.

(15) $$\begin{array}{c} X_{input}=\left[\begin{array}{c} x_{1}^{1}\cdots x_{1}^{f}\\ \vdots \ddots \vdots \\ x_{n}^{1}\cdots x_{n}^{f} \end{array}\right]\text{.} \end{array}$$

The input data first enter the Conv1D layer. A convolution kernel with a convolution window of length *k* is defined as shown in the following equation.

(16) $$\begin{array}{c} f_{k}=\left[\begin{array}{c} w_{1}^{1}\cdots w_{k}^{f}\\ \vdots \ddots \vdots \\ w_{k}^{1}\cdots w_{k}^{f} \end{array}\right],k\leq n-1\text{.} \end{array}$$

In the TensorFlow framework, Conv1D convolutes from top to down. When performing the convolution calculation, a matrix of data fragments of length *k* and width *f*, defined as *X*_*c*_ (17), is first intercepted in the data.

(17) $$\begin{array}{c} X_{c}=\left[\begin{array}{c} x_{c}^{1}\cdots x_{c}^{f}\\ \vdots \ddots \vdots \\ x_{c+k-1}^{1}\cdots x_{c+k-1}^{f} \end{array}\right],c+k-1\leq n\text{.} \end{array}$$

Then, the computational procedure for convolution to generate an output *X*_*f*_ is shown in the following equation.

(18) $$\begin{array}{c} X_{f}=w_{1}^{1}*x_{c}^{1}+w_{1}^{2}*x_{c}^{2}+\cdots +w_{k}^{f}*x_{c+k-1}^{f}\text{,} \end{array}$$

where *l* denotes the convolution kernel size, *p* denotes the use of boundary padding, and *s* denotes the convolution step size. Then, the dimension of the time step after convolution is calculated as shown in the following equation.

(19) $$\begin{array}{c} n_{1}=\frac{n-l+2p}{s}+1\text{.} \end{array}$$

The equation given shows the process of computing the 1D convolution. The above operation is performed on the input matrix using different filters to obtain the output matrix of the convolution layer, where the number of rows of the matrix is *n*_1_ and the number of columns is filers. Next, the operation is continued on the output of the Conv1D layer, which is used as the input of the BiGRU layer. The specific calculation procedure of the BiGRU layer is shown in Sections 2.4 and 2.5 Define *F*_*Conv1D*_ as the Conv1D layer function, *F*_*BiGRU*_ as the BiGRU layer function, *F*_*fc*_ as the fully connected layer function, and *Y*_*pre*_ as the model output. The *Y*_*pre*_ calculation equation is shown in the following equation.

(20) $$\begin{array}{c} Y_{pre}=F_{fc}\left(ReLU\left(F_{BiGRU}\left(ReLU\left(F_{Conv1D}\right)\right)\right)\right)\text{,} \end{array}$$

where *ReLU* (rectified linear unit) is the activation function, which can suppress gradient disappearance and speed up the training speed. In the model training process, the minimum loss function is set as the optimization objective, and then the filter value of the Conv1D layer and the unit value of the BiGRU layer are determined. After that, the number of random seeds, learning rate, and batch size are given for the initialization of the network. Finally, the Adam (adaptive moment estimation) optimization algorithm is applied to continuously update the network weights, and then the final hidden layer network is obtained. To summarize, the above is the formula and principle of the model combining Conv1D and BiGRU. Next, the setting of hyperparameters of the model and the process of using this model for prediction will be introduced in more detail.

### 3.2. GA for Hyperparameter Optimization

Genetic algorithm (GA) is an artificial intelligence-seeking optimization method simulating natural evolution. Furthermore, it is ideal for real-time processing and easy to implement with strong robustness. At present, GA has been successfully applied to various optimization problems [25]. Drawing on the theory of biological evolution, GA models the problem as a biological evolutionary process. It generates the next generation of solutions through operations such as genetics, crossover, mutation, and natural selection. Then, the solutions with low fitness function values are eliminated gradually and those with high fitness functions are increased. In this way, individuals with high fitness will likely be evolved after *N* generations of evolution. The application of GA in neural networks is reflected in three main aspects: learning of networks, structural design of networks, and analysis of networks [26]. In terms of network learning, GA can be used to optimize the learning rules and network weight coefficients. In the structural design of the network, GA can optimize the number of layers, the number of neurons per layer, and the interconnection method of each layer. In terms of network analysis, GA can perform functional analysis, property analysis, and state analysis of neural networks [27]. Here GA is used to perform hyperparameter tuning for the model proposed in the previous section. The common process of GA is shown in Algorithm 1.

The methods of chromosome selection mainly include the roulette selection method, random competitive selection, uniform sorting, and so on. The most used roulette selection method is used here. The methods of gene encoding mainly include binary encoding method, floating-point encoding method, symbolic encoding method, and so on. The binary encoding method is chosen which is easier to decode and encode. In GA, the problem to be solved is mapped into a mathematical problem at first. Then, a feasible solution to this problem is called a chromosome. A feasible solution generally consists of multiple elements, each of which is called a gene on the chromosome. The ultimate goal is to find the chromosome with the best fitness [28]. The process of combining the GA and Conv1D-BiGRU model is shown in Figure 9.

## 4. Experiments

This section describes the dataset and evaluation performance metrics for conducting experiments. Then, the process of hyperparameter search for the proposed model using GA is introduced. Finally, the prediction performance is compared with several models such as LSTM, GRU, BiGRU, and Conv1D-BiLSTM.

### 4.1. Datasets and Performance Metrics

The dataset used in the experiment is from a smelter in Jiangxi Province, China. The dataset consists of 11520 sets of the inlet guide vane position feedback, inlet flow rate, inlet pressure, and outlet pressure data of sulfur dioxide blowers collected every minute from May 1 to May 8 in 2021, as shown in Figure 10. Some data are shown in Table 1. 10,080 sets are used as training sets and valid sets, and 1440 sets are used as test sets. Before the experiment, the datasets need to be split and normalized.

In this experiment, *RMSE* (root mean square error), *MAE* (mean absolute error), and *R*^*2*^ (*R*^*2*^ score) are used as indicators of predictive performance with the following equations.

(21) $$\begin{array}{c} RMSE=\sqrt{\frac{1}{m}\overset{m}{\underset{i=1}{\sum }}{\left(\hat{y_{i}}-y_{i}\right)}^{2}}\text{,} \end{array}$$

(22) $$\begin{array}{c} MAE=\frac{1}{m}\overset{m}{\underset{i=1}{\sum }}\left|\hat{y_{i}}-y_{i}\right|\text{,} \end{array}$$

(23) $$\begin{array}{c} R^{2}=1-\frac{\sum_{i=1}^{m}{\left(\hat{y_{i}}-y_{i}\right)}^{2}}{\sum_{i=1}^{m}{\left(\hat{y_{i}}-y_{i}\right)}^{2}}\text{,} \end{array}$$

(24) $$\begin{array}{c} e_{i}=y_{i}-\hat{y_{i}}, \end{array}$$

where *m* is the number of test samples, *y*_*i*_ and $\hat{y_{i}}$ denote the predicted value and true value, respectively, *y* denotes the mean of the true data, and *e*_*i*_ is the residual of the prediction.

### 4.2. Hyperparameter Optimization

The Conv1D-BiGRU model constructed above involves numerous hyperparameters, the most important of which are the values of filters in the Conv1D layer, the values of units in the BiGRU layer, the learning rate, and batch size. These four hyperparameters are treated as four genes of one chromosome in the genetic algorithm. Among them, the values of filters in the Conv1D layer values are chosen in [16, 32, 64, 128], and unit values are chosen in [16, 32, 64, 128] for BiGRU layer. Learning rate is chosen in [0.1, 0.01, 0.001, 0.0001], and batch size is chosen in [16, 32, 64, 128]. The four genes were binary coded and then randomly combined to generate 20 chromosomes to form the initial population. The probability of crossover between genes in the population was set to 0.7. The probability of variation was set to 0.01. The number of population evolution was set to 20. *T*_*f*_ was set to 0.9. Meanwhile, the fitness function was set as the sum of *RMSE* and *MAE*. The smaller the fitness function was, the better the chromosome was. The result of the evolution of the population after 20 generations is shown in Figure 11.

Figure 10 shows that the smallest value of the fitness function is found for a chromosome of [64, 128, 0.001, 64] in 20 generations of population evolution, where the *RMSE* is 0.504 and the *MAE* is 0.406. At this time, the four hyperparameters and other parameters of the model determined using this excellent chromosome were set as shown in Table 2.

The prediction results of Conv1D-BiGRU using the parameters obtained by GA in Table 3 are shown in Figure 12.

### 4.3. Prediction Performance Comparison with Other Models

To verify the accuracy of the prediction of the proposed model, it is compared with the LSTM, GRU, BiLSTM, BiGRU, and Conv1D-BiLSTM models. The prediction accuracy of these models is evaluated on the test set using the three metric evaluation criteria presented in the previous section. The hyperparameter set is used in Section 4.2, and the evaluation results of the different models are shown in Table 3. The prediction error is shown in Figure 13. Table 3 and Figure 13 show that the model combining Conv1D and BiGRU outperforms the LSTM, GRU, BiLSTM, BiGRU, and Conv1D-BiLSTM models for time series data, and the proposed model in terms of evaluation metrics performs the best.

After the experimental comparison, the proposed model has the best effect on the outlet pressure prediction of the sulfur dioxide blower after the GA optimization. Table 3 shows that the model has the best performance among the three evaluation indexes, and Figure 13 shows that the prediction residual curve of the model has a small and flat fluctuation range.

## 5. Conclusions

The monitoring of the outlet pressure of the sulfur dioxide blower in the process of acid production with flue gas is crucial. To achieve early warning of the abnormal outlet pressure of the sulfur dioxide blower, a model combining Conv1D-BiGRU and GA is proposed. Compared with the structure of other prediction models, Conv1D can well integrate the information between different variables and mine the correlation features and periodic features among them, while BiGRU can observe the information of blower in different periods and learn the time series relationship of the features extracted by Conv1D. As a result, it can well deal with the complexity and nonlinearity of time series data. The combination of the two models can capture not only the correlation information of the coupling relationship between variables on the spatial scale but also the development trend between variables on the temporal scale. Importantly, GA is used to find the optimization of important hyperparameters in the construction and training of the Conv1D-BiGRU model, which largely improves the performance of the model.

The model is validated using real historical data of a sulfur dioxide blower in a smelter in Jiangxi Province. First, the data of variables highly correlated with the outlet pressure are selected for data processing based on the relevance and operation mechanism of the sulfur dioxide blower. After that, the Conv1D-BiGRU model is used to capture the variable coupling relationship on the spatial scale and the development trend on the temporal scale of the variables. The value of the outlet pressure is predicted by the proposed model. Finally, the important parameters of the Conv1D-BiGRU model are tuned and set using GA to improve the accuracy of pressure prediction. The combination of the Conv1D-BiGRU model and GA can make an accurate prediction of the outlet pressure of the sulfur dioxide blower in the short term and provide early warning of abnormal working conditions, which can help plants to make process adjustments and increase production efficiency. In the subsequent research work, an attention mechanism will be considered to predict exit pressure in conjunction with the above methods.

## Figures and Tables

**Figure 1:** System architecture.

**Figure 2:** Sulfur dioxide blower (from Guixi Smelter, Jiangxi Province, China).

**Figure 3:** The process of acid production with flue gas.

**Figure 4:** CNN structure.

**Figure 5:** LSTM cell structure.

**Figure 6:** GRU cell structure.

**Figure 7:** BiGRU cell structure.

**Figure 8:** Model structure.

**Figure 9:** GA-Conv1D-BiGRU structure.

**Figure 10:** Variable sequence diagram. (a) Inlet guide vane position (%). (b) Inlet pressure (kPa). (c) Inlet flow rate (Nms/h). (d) Outlet pressure (kPa).

**Figure 11:** Population evolution.

**Figure 12:** Prediction results.

**Figure 13:** Prediction residual of different models.

**Algorithm 1:** GA.

**Table 1:** Partial data display.

Sets	…	100	101	…	10000	10001	…
Inlet guide vane position (%)	…	12.54108429	12.53520871	…	23.13002205	23.12452698	…
Inlet pressure (kPa)	…	−6.05723142	−6.03437233	…	−6.37186288	−6.37623786	…
Inlet flow rate (Nms/h)	…	127830.9141	128445.0625	…	163426.7813	161879.8125	…
Outlet pressure (kPa)	…	25.43690491	25.53358841	…	35.24561691	35.10400773	…

**Table 2:** Parameter setting.

Filters of Conv1D	64
Units of BiGRU	128
Learning rate	0.001
Batch size	64
Dropout rate	0.2
Epochs	100

**Table 3:** Comparison of prediction accuracy of different models.

Model	Criteria		
	RMSE	MAE	*R * ^2^
LSTM	0.610	0.507	0.990
GRU	0.626	0.495	0.990
BiLSTM	0.618	0.487	0.991
BiGRU	0.621	0.484	0.988
Conv1D-BiLSTM	0.575	0.457	0.992
Conv1D-BiGRU	0.504	0.406	0.993

## Data Availability

The datasets used and analyzed during the current study are available from the corresponding author upon reasonable request.
